# Downregulation of miR-221-3p by LncRNA TUG1 Promoting the Healing of Closed Tibial Fractures in Mice

**DOI:** 10.1155/2022/1624446

**Published:** 2022-08-26

**Authors:** Laiyou Liu, Yinpeng Yuan

**Affiliations:** Department of Orthopedics, The Second Hospital of Shanxi Medical University, Taiyuan, 030001 Shanxi, China

## Abstract

**Objective:**

To probe into the effect of LncRNA TUG1 on the healing of closed tibial fracture in mice.

**Methods:**

The closed tibial fracture model of mice was established, selecting the mouse osteoblast line MC3T3-E1, with the cells separated into four groups. The expression levels of TUG1 and miR-221-3p were determined by RT-qPCR analysis, with the targeting relationship between TUG1 and miR-221-3p authenticated by dual luciferase reporter (DLR) assay, detection of cell migration (CM) ability based on Transwell cell migration (TCM) assay, and cell proliferation (CP) acquired by cell counting kit-8 (CCK-8).

**Results:**

Prediction results of the target gene by bioinformatics software showed that miR-221-3p had binding sites with the 3′-UTR of TUG1, and DLR assay authenticated the targeting relationship between LncRNA TUG1 and miR-221-3p. Downregulation of TUG1 inhibited osteoblast CP and CM and promoted osteoblast cell apoptosis (CA). Cell cycle analysis indicated that miR-221-3p provoked cell cycle arrest in G1 stage of MC3T3-E1 cells. The siLncRNA-NC group had higher anticyclin D1 and D3 levels than the siLncRNA TUG1 group, with a lower CA rate in the former, implying that miR-221-3p overexpression inhibited osteoblast CP and CM and LncRNA TUG1 inhibited CA. Downregulation of miR-221-3p partly reversed the retardation out of downregulating TUG1 on osteoblast CP and CM. Bcl-2 level was higher in the LncRNA TUG1 group compared to the siLncRNA TUG1 and miR-221-3p overexpression groups, with remarkably lower SDF-1 level in the miR-221-3p overexpression group than those in the control, miRNA-NC, and LncRNA TUG1 groups.

**Conclusion:**

The downregulation of miR-221-3p by LncRNA TUG1 can promote the healing of closed tibial fractures in mice.

## 1. Introduction

Fracture healing is a complex natural recovery process after the occurrence of traumatic fractures with the involvement of multiple molecules and cells among which osteoblast cell proliferation (CP) and cell apoptosis (CA) play a pivotal part in bone healing and remodeling [1]. MicroRNAs (miRNAs), as single-stranded, endogenous, noncoding small RNA molecules, can bind with the 3′-untranslated region (3′-UTR) of target messenger RNAs and affect the differentiation and growth of osteoblasts, chondrocytes, and osteoclasts. According to related studies, LncRNA TUG1, a chromatin-modifying complex located on human chromosome 22q12.2, has a high expression in vascular endothelial cells and regulates the CP and CA of oncocytes, making it a potential tumor biomarker and therapeutic target [2]. Currently, a lot of research has authenticated that LncRNA TUG1 influences the malignant behavior of tumors by inhibiting miRNAs [3, 4]. For instance, LncRNA TUG1 can adsorb miR-29c-3p, which enhances the malignant behavior of gastric adenocarcinoma [5]. Yao et al. have found that knockout of LncRNA TUG1 can inhibit viability, CM, and differentiation and lead to CA of osteoblasts in patients with maxillary fractures, suggesting that LncRNA TUG1 is also involved in the biological process of osteoblast CP and CA [6].

Inhibitory miRNAs can inhibit osteoblast CP and promote CA by targeting osteogenic genes in vitro [7, 8]. For example, increased miR-221-3p expression during bone healing in diabetic fracture patients can lead to impaired endochondral ossification and reduced bone remodeling [9]. miR-221-3p, a member of miR-221, can regulate the CP and differentiation of oncocytes in gastric, thyroid, and hepatic cancers. This miRNA has an approximate mechanism in bone healing in patients with osteoarthritis, and because of its mechanosensitivity, extracellular vesicles in chondrocytes of osteoarthritis patients can transfer it to osteoblasts so that it acts as an intercellular messenger to reduce the bone formation of osteoblasts in vitro [10]. Although no studies have analyzed the function of miR-221-3p on closed tibial fracture patients, the discovery of this miRNA undoubtedly provides information on the pathological process of bone healing in closed tibial fracture patients. Since the targeting relationship with miR-221-3p and ability of adsorbing miRNA and partly reversing its retardation effect, the analysis of long-noncoding RNA (LncRNA) is expected to offer an innovative strategy for treating closed tibial fracture patients. There is still a gap in the research of LncRNA TUG1 and miR-221-3p affecting closed tibial fractures, so this study will explore the molecular mechanism of LncRNA TUG1 promoting osteoblast CP and CM in closed tibial fractures through downregulation of miR-221-3p.

## 2. Materials and Methods

### 2.1. Fracture Model of Animal

SPF 5-6-week-old BALB/c mice (*n* = 60) (Beijing Vital River Laboratory Animal Tech. Co., Ltd.; SCXK (Jing)-2016-0011) were fed in the IVC system of the Animal Experimental Center. The research conformed to the standards of the Animal Care and Use Review Office, and relevant operations were implemented based on the animal management regulations of SSTC of China. Anesthesia was performed with 3% isoflurane (Lunanbeite Pharma. Co., Ltd., CN). A sterile bench was established for posterolateral incision and blunt dissection of the right tibial fracture model of mice before disinfecting by 0.5% povidone iodine solution (Nanda Pharma. Co., Ltd., Nanjing, CN). The tibia was cut with a diamond disc, with the fracture site fixed with a 0.6 mm intramedullary needle. 30 mice were executed on day 14 after fracture to obtain samples for in-depth analysis, with the remaining mice executed in subsequent experiments.

### 2.2. Treatment of Mice in Fracture Model

On days 0, 4, and 7 after surgery, 100 *μ*L of fetal bovine serum (FBS) (Thermo Fisher Sci., SH, CN) was applied to the fracture site of mice in the control group, with 100 *μ*L of 200 *μ*M FBS applied to the siLncRNA TUG1 group, LncRNA TUG1 group, and simiR-221-3p group.

### 2.3. Cell Culture and Transfection

MC3T3-E1, from the cell bank of CAS, was chosen as the murine osteoblastic cell lines. They were cultured in an incubator (37°C, 5% CO_2_) with *α*-MEM (Thermo Fisher Sci., SH, CN) (containing 10% FBS (Thermo Fisher Sci., SH, CN) and 1% Pen/Strep (Pfizer, NY, USA)) and dissociated with 0.25% trypsin (Thermo Fisher Sci., SH, CN), with cell passage followed. The logarithmic growth phase cells in good condition were used for subsequent experiments. LncRNA TUG1-NC, LncRNA TUG1, and simiR-221-3p were synthesized artificially by a gene pharmaceutical company (Sanyuan Gene Pharma. Co., Ltd., Beijing, CN) under the condition of 200 *μ*M FBS and transfected into MC3T3 cells with Lipofectamine™ 3000 transfection reagent (Invitrogen, CA, USA). All operations were performed strictly based on the instructions, with a 48 h of incubation of the transfected cells for RNA and protein analysis.

### 2.4. CCK-8 Assay

Before 4 h of incubation at 37°C, the cells were planted in 96-well plates (1 × 10^3^ cells/well), supplemented with 10 *μ*L of CCK-8 solution. The number of viable cells was detected indirectly by a microplate reader (German Railway Testing Equip. Co., Ltd., Nanjing, CN).

### 2.5. Apoptosis Assay

Before the analysis on cycle status by the cell cycle assay kit (KeyGEN BioTECH, Jiangsu, CN), the cells were planted in 6-well plates (1 × 10^6^ cells/well) with a 48 h transfection. They were separated and fixed in 70% ice-cold ethanol at room temperature of 4°C overnight and then rinsed by PBS and marked by 500 *μ*L of reaction solution (RNAse/PI = 1/9) for 30 min. Later, the cells were analyzed using ModFit LT of a flow cytometer (FACS Calibur American BD Company, USA), with the CM of MC3T3-E1 cells assessed by Annexin V-FITC/PI apoptosis assay kit (BD Company, USA). Briefly, the treated cells were rinsed with ice-cold PBS and resuspended in 500 *μ*L BB, and then, they were processed with 5 *μ*L of Annexin V-FITC and 5 *μ*L of PI for 15 min in a dark condition and kept at room temperature, with analysis of flow cytometer.

### 2.6. TCM Assay

Resuspend the cells (1.5 × 10^4^cells/well) in a low-serum (5% FBS) medium, which were planted into the upper chamber of a 24-well Transwell plate (Corning, Corning, NY, USA) containing an 8 *μ*m pore size filter, with the lower chamber as a complete medium with 10% FBS for compound testing. The cells migrating to the bottom surface were dyed by 0.5% CrV and observed microscopically (Topcon Co., Ltd., Japan) after 12 h, with those on the upper surface of the filter membrane rinsed.

### 2.7. Dual Luciferase Reporter (DLR) Assay

The wild sequence (WT) and mutant sequence (MUT) for the synthesis of TUG1 3′-UTR were designed and amplified, and the amplified fragments were transferred into the miRNA expression vector (Applied Biosystems) of pMIR-reporterTM to construct recombinant plasmids capable of expressing luciferase. The constructed recombinant plasmids were transfected into MC3T3-E1 cells together with miR-221-3p mimics and miRNA-NC. After 72 h, the cells were collected, with the procedure performed in strict line with the directions of luciferase reporter gene assay kit. Finally, the ratio of firefly fluorescence to Renilla fluorescence was measured by a chemiluminometer to analyze the binding force between miR-221-3p and TUG1.

### 2.8. RT-qPCR Analysis

The cells were processed with TRIzol reagent (Thermo Fisher Sci., SH, CN), with RNA concentration and purity determined by ultra-micronucleic acid quantitation spectrometer (Thermo Nanodrop 1000). The reverse transcription was implemented based on the directions from the cDNA reverse transcription kit (All-in-One™ miRNA First-Strand cDNA Synthesis Kit), with 2 *μ*g RNA taken for reverse transcription into cDNA per sample for RT-qPCR detection. Reaction conditions are as follows: 30 s of predenaturation at 95°C, followed by 40 cycles of 95°C for 5 s and 60°C for 30 s. With U6 of each sample as an internal reference, the relative gene expression was calculated and analyzed by the 2^-*ΔΔ*Ct^ method, with the primer sequences detailed as Table 1.

### 2.9. Immunoblot Analysis

Extraction of total cellular protein was achieved by lysing the cells in RIPA buffer and washing them with PBS, with the lysates placed in 10% SDS-PAGE and proteins transferred to PVDF membranes (Millipore, Schwalbach, Germany). The cytomembranes were mainly probed with anticyclin D1 and D3 (1 : 1000, Yansheng Biochemical Reagent, SH, CN), with protein bands observed by chemiluminescence (Canon, Tokyo, Japan, #LiDE110) before incubation with appropriate secondary antibodies.

### 2.10. Statistical Disposal

The data were processed mainly by SPSS 20.0, with the measurement data represented as mean ± std.deviation ($\overset{¯}{x}\pm s$). The statistical methods used included one-way ANOVA and *t*-test. The graphs were plotted with GraphPad Prism 6. *P* < 0.05 indicated a statistically remarkable difference.

## 3. Results

### 3.1. Targeting Relationship between LncRNA TUG1 and miR-221-3p

Target genes were predicted by bioinformatics software such as microRNA.org, TargetScan, and miRBase, with results showing that miR-221-3p had binding sites with 3′-UTR of TUG1 (Figure 1(a)). DLR assay suggested that in contrast to the miRNA-NC group, the miR-221-3p group had a decreased luciferase activity in WT-TUG1 cells, while that in MUT-TUG1 cells was not affected (Figure 1(b)). Further research revealed the decreased miR-221-3p expression of the LncRNA TUG1 group in contrast to the control and siLncRNA-NC groups (Figure 1(c)).

### 3.2. Downregulation of TUG1 Inhibited CP and CM and Promoted CA of Osteoblasts

On the basis of CCK-8 and TCM assays, no remarkable change was found at 24 h in the cell viability of all groups (*P* > 0.05), with remarkably lower cell activity in the siLncRNA TUG1 group than those in the control and siLncRNA-NC group at 48 h and 72 h (*P* < 0.001). It was revealed that compared to siLncRNA-NC, siLncRNA TUG1 significantly inhibited CP and CM (Figures 2(a) and 2(b)). According to cell cycle analysis, anticyclin D1 and D3 levels were higher in the siLncRNA-NC group than in the siLncRNA TUG1 group (Figure 2(c)). Compared to the siLncRNA TUG1 group, the CA rate was lower in the siLncRNA-NC group, whose cells were dyed by Annexin V-FITC and PI (Figure 2(d)).

### 3.3. Overexpression of miR-221-3p Inhibited Osteoblast CP and CM

The results of CCK-8 and TCM assays showed that the miR-221-3p level remarkably increased in MC3T3-E1 cells of the miR-221-3p overexpression group compared to the miRNA-NC group, suggesting the successful construction of miR-221-3p-overexpressing MC3T3-E1 cell line. The viability of MC3T3-E1 cells of the miR-221-3p overexpression group did not change remarkably at 24 h and was remarkably lower than those in the control group and miRNA-NC group at 48 h and 72 h (Figure 3(a)), confirming that overexpression of miR-221-3p inhibited CP, and the CM ability was also lower than those in the control and miRNA-NC groups (Figure 3(b)). Cell cycle analysis also revealed that its anticyclin D1 and D3 levels were remarkably lower than those in the miR-NC and control groups (Figure 3(c)). In addition, Annexin V-FITC and PI staining showed that the miR-221-3p overexpression group had a high CA rate (Figure 3(d)).

### 3.4. Downregulation of miR-221-3p Partly Reversed the Retardation out of Downregulating TUG1 on Osteoblast CP and CM

Compared to the siLncRNA TUG1 group, the cell viability of MC3T3-E1 in the siLncRNA TUG1+simiRNA group did not change remarkably at 24 h and increased remarkably at 48 h and 72 h (Figure 4(a)), with distinctly increased CM number of MC3T3-E1 (Figure 4(b)). The above results authenticated that downregulation of miR-221-3p partly reversed the retardation out of downregulating TUG1 on osteoblast CP and CM.

### 3.5. Downregulation of LncRNA TUG1 Inhibited Closed Tibial Fracture Healing in Mice

Bcl-2, an antiapoptotic signaling protein in the downstream of P53, acts as a pivotal part in regulating CA. Compared to the siLncRNA TUG1 and miR-221-3p overexpression groups, the Bcl-2 level in the LncRNA TUG1 group was higher (Figure 5). SDF-1 was a protein involved in bone regeneration and bone repair. The SDF-1 level in the miR-221-3p overexpression group was remarkably lower than those in the control, miRNA-NC, and LncRNA TUG1 groups (Figure 5). The above results revealed that miR-221-3p obstructed the healing of closed tibial fractures in mice, and the downregulation of LncRNA TUG1 played the same role.

## 4. Discussion

LncRNA is a noncoding RNA with a transcript of >200 nt in length, which can perform biological functions as an important class of regulatory molecules in the human genome and coordinate the complex regulatory processes of higher life [11–13]. Recent research has shown that LncRNAs can also act as a competitive endogenous RNA to form double-stranded RNA with complementary miRNA, which can affect the processes of miRNA splicing, processing, and translocation, and participate in the expression of target genes, thus influencing CP, differentiation, and CA [1, 14]. Currently, the academic community has a mature understanding of the regulatory mechanisms of anti-oncogene-related ceRNA, but there is a relative lack of ceRNA studies on fracture healing. With the changing lifestyles of Chinese residents, the incidence of fractures is gradually increasing, as well as the number of patients with closed tibial fractures, including both patients with severe closed tibial fractures due to high-energy damage and elderly patients with osteoporotic closed tibial fractures due to low-energy damage [15–17]. Deepening the research on LncRNA and miRNA can offer important insights into the biological process of bone and bone healing and provide new ideas for treating closed tibial fractures clinically.

At present, some LncRNAs functioning in osteoblast CP, CM, and CA have been demonstrated; for instance, Huang et al. have found that LncRNA H19 can play an important part in osteoblast differentiation through the TGF-*β*1/Smad3/HDAC signal path [18]. Yu et al. have reported that LncRNA HOXA11-AS can adsorb miR-124-3p to accelerate osteoblast CA. LncRNA TUG1 has been less studied in bone healing, but a study has shown that it can adsorb miR-204-5p, which can upregulate RUNX in aortic valve calcification and accelerate osteoblast differentiation [19]. Another study has shown that LncRNA TUG1 can influence osteoblast CP and differentiation through the Wnt/*β*-catenin signal path [20]. Based on the above studies showing an increase in LncRNA TUG1 during fracture healing, this study assumes that LncRNA TUG1 plays a promoting role in fracture healing. To this end, the healing tissue models of intact control bone and closed tibial bone in mice with differential expression of LncRNA TUG1 were constructed, with the performance of a DLR assay confirming the targeting relationship between LncRNA TUG1 and miR-221-3p. For purpose of in-deep research on the molecular mechanism of these two in CP, CM, and CA of MC3T3-E1 cells, CCK-8 and TCM assays were carried out. It was found that downregulation of LncRNA TUG1 restricted the CP and CM of MC3T3-E1 cells and supported their CA, while overexpression of miR-221-3p inhibited osteoblast CP and CM, which was reversed in the miRNA-NC group. In contrast to the miR-221-3p overexpression group, CP rate in the miRNA-NC group remarkably increased after transfection. Flow cytometry revealed that the MC3T3-E1 cell cycle progressed from G0/G1 to S, G2/M in this group, and G1/S transition was hindered by overexpression of miR-221-3p. As for the miR-221-3p overexpression group, the anticyclin D1 and D3 levels were also remarkably reduced, with a higher CA rate corroborated by Annexin V-FITC, confirming that miR-221-3p promoted CA of MC3T3-E1 cells.

Further study revealed that compared with siLncRNA TUG1 and miR-221-3p overexpression groups, the Bcl-2 level in the LncRNA TUG1 group was higher, with remarkably lower SDF-1 level in the miR-221-3p overexpression group than those in the control, miRNA-NC, and LncRNA TUG1 groups. SDF-1, a part of the *α* chemokine family, whose specific receptor CXCR4 is expressed on the surface of many cells, and the two can constitute the SDF-1/CXCR4 axis, serving as a key part in tissue injury and bone damage repair [21–23]. Clinical studies have shown that the secretion of SDF-1 in the bone repair site increases, and CXCR4+-committed stem cells around bone marrow, peripheral circulating blood, and soft tissue of bone trauma migrate to the bone injury site along the gradient of SDF-1 concentration to participate in bone healing [24]. Kawakami et al. have reported that the SDF-1/CXCR4 axis in Tie2-spectrum cells, which includes EPCs, accelerates fracture healing [25], while the study of Arakura et al. showed that SDF-1 levels were remarkably lower during fracture healing in diabetic patients than in the healthy group, suggesting that differential gene expression of SDF-1 is one of the reasons for poor fracture healing in diabetic patients [26]. Moreover, SDF-1 is also closely related to angiogenesis, the high expression of which indicates good blood supply, bringing necessary environmental nutritional support for bone regeneration [27]. Therefore, the low SDF-1 level in the miR-221-3p overexpression group implies that the fracture site is accompanied by tissue ischemia and hypoxia, and endochondral ossification is thus affected. Zheng et al. stated that downregulating miR-221-3p directly targeted the SDF1/CXCR4 signal path and promoted IL-1*β*-induced cartilage degradation, confirming that cartilage degeneration grade correlates with miR-221-3p level, and that the protection of miR-221-3p against chondrocyte extracellular matrix degradation proceeded through SDF1/CXCR4 signal transduction [28]. Since LncRNA can compete with target gene mRNA to bind miRNA response elements, inhibit miRNA expression, and indirectly increase the expression level of target genes, LncRNA TUG1 can inhibit the retardation effect of miR-221-3p on osteoblast CP and CM; i.e., downregulation of miR-221-3p can partly reverse the retardation out of downregulating TUG1 on the CP and CM of osteoblasts.

In this study, no clinical trial was conducted to probe into the effect of LncRNA TUG1 in closed tibial fracture patients. In summary, the study clarifies the adsorption capacity of LncRNA TUG1 on miR-221-3p and confirms that downregulation of miR-221-3p by LncRNA TUG1 promotes the healing of closed tibial fractures.

## Figures and Tables

**Figure 1:** (a) Targeting relationship between LncRNA TUG1 and miR-221-3p. (b) TUG1 expression levels acquired by DLR assay. (c) miR-221-3p expression levels acquired by RT-qPCR assay; ^∗^*P* < 0.001.

**Figure 2:** (a) CM acquired by TCM assay. (b) CP acquired by CCK-8 assay. (c) Anticyclin D1 and D3 levels based on immunoblot analysis. (d) CA rates acquired by apoptosis assay; ^∗^*P* < 0.001.

**Figure 3:** (a) CM acquired by CCK-8 assay. (b) CP acquired by TCM assay. (c) Anticyclin D1 and D3 levels based on immunoblot analysis. (d) CA rates acquired by apoptosis assay; ^∗^*P* < 0.001.

**Figure 4:** (a) CP acquired by CCK-8 assay. (b) CM acquired by TCM assay; ^∗^*P* < 0.001.

**Figure 5:** Protein expression levels based on immunoblot analysis; ^∗^*P* < 0.001.

**Table 1:** qPCR primer sequence (5′→3′).

Genes	Sequences
miR-221-3p	Forward primer 5′-ACACTCCAGCTGGGAGCTACATTGTC-3′
	Reverse primer 5′-CTCAACTGGTGTCGTGGA-3′

TUG1	Forward primer 5′-TCAGTAGCTGCCACCATG-3′
	Reverse primer 5′-TGCTTGGTGAGTCGTGTCTC-3′

U6	Forward primer 5′-AGAGAAGATTAGCATGGCCCCTG-3′
	Reverse primer 5′-ATCCAGTGCAGGGTCCGAGG-3′

## Data Availability

Data to support the findings of this study is available on reasonable request from the corresponding author.
